# Circular RNA SMARCA5 Modulates Epithelial-Mesenchymal Transformation, Proliferation, and Metastasis of Nasopharyngeal Carcinoma Cells via microRNA-582-3p/Phosphatase and Tensin Homolog Axis

**DOI:** 10.1155/2023/5177471

**Published:** 2023-01-13

**Authors:** Hui Wang, HaiTang Ren

**Affiliations:** Department of Otorhinolaryngology, Tianjin Hospital, Tianjin 300000, China

## Abstract

The action mechanism in which circular RNA (circ) SMARCA5 targeted nasopharyngeal carcinoma (NPC) cell proliferation, migration, invasion, and apoptosis via microRNA (miR)-582-3p/phosphatase and tensin homolog (PTEN) axis was explored. The examination was performed via reverse transcription-quantitative polymerase chain reaction (RT-qPCR), discovering that circSMARCA5 was elevated while miR-582-3p was silenced in NPC tissues and cells. E-cadherin and N-cadherin were detected. The results illustrated transfection with si-circSMARCA5 or miR-582-3p-mimic was available to repress cancer cell advancement, and E-cadherin was augmented. Transfection with pcDNA 3.1-circSMARCA5 or miR-582-3p-inhibitor was available to accelerate cancer cell advancement, and N-cadherin was augmented. MiR-582-3p-inhibitor blocked the suppression of si-circSMARCA5 on NPC. The si-PTEN blocked the malignant behavior of pcDNA 3.1-circSMARCA5 against NPC. The binding sites between circSMARCA5 and miR-582-3p and between miR-582-3p and PTEN were verified. Linear analysis results illuminated the expression pattern of circSMARCA5 was opposite to miR-582-3p, while the expression pattern of circSMARCA5 was positively associated with PTEN. In brief, the results of the research clarified circSMARCA5 modulated NPC cells' vital movement via the miR-582-3p/PTEN molecular axis.

## 1. Introduction

Nasopharyngeal cancer (NPC) is caused by the dysfunction of nasopharyngeal epithelial cells [1]. The illness is the popular head and neck malignant tumor in China, and the incidence rate in Guangdong is the highest at about 0.7‰. Early NPC normally occurs in hidden locations, like the pharynx's indentation and the roof, which makes it hard for people to detect, so numerous NPC patients have deteriorated to the advanced stage when they see a doctor [2]. Radiotherapy has a definite efficacy on NPC [3], but drug tolerance during radiotherapy is available to hinder NPC's prognosis [4]. Consequently, it is critical to identify biomarkers for altering NPC's occurrence and development.

Circular RNA (circRNA) is a circular gene derived from reverse splicing of protein encoding. It outweighs linear RNA in indicating pathological or physiological changes in organisms, and circRNA has high stability and a long half-life [5]. With the advancement of science and technology, circRNA's action has drawn numerous attention. For instance, ciRS-7 implicates in tongue squamous cell carcinoma's pathogenesis and interacts with miR-7 to slow down cancer cell proliferation [6]. CircAMOTL1 impacts the progression of cervical cancer (CC) via a competitive combination of miR-485-5p [7]. CircSMARCA5, as a member of circRNA, has also been discovered to be associated with numerous cancers. For instance, circSMARCA5 is available to suppress prostate cancer (PCa) cell advancement via binding downstream target genes' molecular axis [8]. CircSMARCA5 is a glioblastoma multiforme biomarker [9]. CircSMARCA5 is available to boost osteosarcoma cell advancement with enhancive adhesion via a competitive endogenous RNA network [10]. Nevertheless, the regulatory mechanism of circSMARCA5 in NPC has not been explored and reported.

CircRNA is available to immediately combine with the 3′ untranslated region (UTR) of microRNA (miRNA), adjust miRNA, render messenger RNA (mRNA) to lyse, or restrain target proteins' translation. miRNA is available to modulate cancer cell functions like growth in this way. Consequently, it is critical to illuminate miRNA's action in cancer specificity [11]. Several studies have discovered that miRNAs are available to be adopted as tumor suppressor or cancer-promoting genes. For instance, miR-411-5p is available to restrain PCa's occurrence and development via silencing SMAD3 and TGFBR2 proteins [12]. Fibulin 5 and miR-552-3p can be combined to promote lung cancer (LC) cell growth [13].

Numerous researches have been presented on the modulation of miR-582-3p in cancer, for instance, miR-582-3p is available to target HUR and VEGF proteins to impact gastric cancer (GC) development [14], elevated miR-582-3p is available to repress hepatocellular carcinoma (HCC) tumor formation [15], etc. Meanwhile, miR-582-3p also acts as a sponge target by some long noncoding RNAs. Wang reported lncRNA HOXA10-AS facilitates proliferation and migration of NPC through sponging miR-582-3p to upregulate RAB31 and suggests that miR-582-3p is involved in the disease progression of NPC (PMID: 35072529). Nevertheless, whether circSMARCA5 plays a regulatory role through miR-582-3p in NPC remains to be further explored. Phosphatase and tensin homolog (PTEN) is one of the tumor suppressor genes and is most frequently activated in sporadic cancer (PMID: 21430697). Of note, our sequence analysis and mRNA‐miRNA interaction prediction revealed that PTEN is a potential target gene of miR‐582-3p. Interestingly, the downregulation of PTEN promotes tumor cell growth, migration, and invasion in NPC cells (PMID: 23125220). And on the contrary, enhancing PTEN expression promotes the autophagy and apoptosis of NPC cells (PMID: 33332708). Based on these aforementioned findings, we have suggested an interaction of circSMARCA5 in the biological process via miR-582-3p/PTEN axis.

circSMARCA5 was selected as the research object in this study to explore the role of circSMARCA5/miR-582-3p/PTEN in modulating NPC development mechanisms and action covering epithelial-mesenchymal transition (EMT), proliferation, migration, invasion, and apoptosis to provide new targets and insights for NPC therapy and diagnosis. In recent years, traditional Chinese medicine has had significant efficacy in terms of improvement of quality of life, alleviation of acute adverse effects, and enhancement of immunoregulation in the treatment of NPC compared with general radiotherapy and chemotherapy (PMID: 24965419). For example, *G. glabra* decreased proliferation and induced the apoptosis of NPC cells (PMID: 31066003). The exploration of the mechanism of circSMARCA5 is expected to provide a new perspective on the treatment of traditional Chinese medicine in NPC.

## 2. Materials and Methods

### 2.1. Experimental Subjects

From October 2015 to October 2020, enrollment of 40 patients who were first diagnosed with NPC in Tianjin Hospital was implemented. NPC tissue and matched nontumor tissue (≥3 cm, *n* = 40) were obtained from NPC patients following surgery or biopsy, and the tissues were electroblotted and stored on liquid nitrogen immediately. None of the patients had a history of tumor and did not receive any treatment for NPC. Informed consents were signed by all patients participating in the experiment, and authorization of the experiment's enforcement was from the Medical Department of Tianjin Hospital and its ethics committee.

### 2.2. Experimental Subjects

Human NPC cell lines CNE1, CNE2, and HONE1 and human embryonic nasopharyngeal epithelial cells HENE were purchased from the Chinese Academy of Sciences (Shanghai, China). Dulbecco's modified Eagle medium (DMEM), fetal bovine serum (FBS), 1% penicillin-streptomycin mixture, and 0.2% trypsin were purchased from ThermoFisher (USA). All the cells were cultured in DMEM with 10% FBS and 1% penicillin-streptomycin mixture. 0.2% trypsin was used for the detachment of passage. In subsequent experiments, cells in the logarithmic growth phase were chosen. pcDNA-circSMARCA5, pcDNA3.1, si-circSMARCA5/NC, in/mimic-NC, miR-582-3p-mimic/inhibitor, si-PTEN were purchased from GenePharma (Shanghai, China). On the grounds of the instructions of Lipofectamine™ 2000 kit (Invitrogen, USA), the above plasmids or oligonucleotide was transfected into CNE2 cells. After 48 h, NPC cell lines were collected.

### 2.3. (4,5-Dimethylthiazol-2-yl)-2,5-Diphenyltetrazolium Bromide (MTT) and Cell Colony Formation Assay

In the light of the foregoing research methods, cell proliferation was detected via MTT assay and cell colony formation assay [16, 17]. The cells were seeded in 96-well plates with a density of 1 × 10^5^/well. 25 *μ*L 5 mg/mL of MTT solution (Sigma, USA) was added to each well at 0, 24, 48, 72, and 96 h separately with continuous culture. Then, cells were treated with the addition of 100 *μ*L DMSO solution (Sigma). Each well's absorbance was measured at 490 nm adopting a microplate detector. CNE2 cells in the logarithmic growth phase were seeded into 6-well plates at a density of 800 cells/well. Then, the cells were cultured for 2 to 3 weeks until visible cloned cell clusters appeared in Petri dishes. The colonies were added with 5 ml of the mixture (acetic acid:methanol = 1:3 (analytically pure, Jianxing reagent, Guangzhou)), fixed, and stained with Giemsa staining solution. The surviving cells were counted. The formulas for counting colonies were as follows: colony number = total number of cell colonies in N wells/N and colony formation rate = colony number/total number of cultured cells × 100%.

### 2.4. Transwell Assay

In line with the foregoing researches, cell migration and invasion abilities were tested by Transwell assay [18]. 3 × 10^3^ well-grown CNE2 cells were seeded into the Transwell plate's upper chamber, and the addition of 200 *μ*L serum-free Roswell Park Memorial Institute (RPMI)-1640 medium was implemented, and 600 *μ*L RPMI-1640 medium covering 10% FBS was added into the lower chamber and incubated. Subsequently, fixation and staining were with 4% paraformaldehyde and 0.5% crystal violet (both Aladdin, Shanghai, China). Random selection of nine fields was from each sample and observation was under an optical microscope (×200) to calculate the mean cell number. For the invasive ability test, precoating of each Transwell upper chamber was with 30 *μ*L BD Matrigel matrix (Beijing qualityard biotechnology Co., Ltd). After solidification, hydration of the matrix membrane was with serum-free DMEM (ThermoFisher), and the following steps were the same as mentioned above.

### 2.5. Flow Cytometry

As presented in antecedent researches, CNE2 cell apoptosis is analyzed via flow cytometry [19]. Annexin V-Fluorescein isothiocyanate (FITC)/Propidium iodide (PI) kit (Vazyme, Nanjing, China) was adopted to assess the percentage of apoptotic cells (FITC+/PI±). After 72 h of transfection, 400 *μ*L buffer covering CNE2 cells was taken and staining was with the addition of 5 *μ*L Annexin V-FITC and PI. Apoptosis cells were captured with FITC+/PI± adopting a flow cytometer, and the apoptosis rate was analyzed.

### 2.6. Reverse Transcription-Quantitative Polymerase Chain Reaction (RT-qPCR) Detection

RT-qPCR was performed to detect miRNA and mRNA as mentioned above [20]. The extraction of total RNA was from NPC tissues and cells adopting TRIzol kit (Invitrogen). Then, RNA was reverse transcribed into a complementary DNA (PrimeScript RT Master Mix, Takara, Dalian, China), and amplification was on a real-time PCR instrument. The PCR was accomplished in the light of the instructions in the SYBR Green RT-qPCR kit (Takara). U6 and *β*-actin were adopted as loading control for miRNA and mRNA, respectively. The adoption of 2^−ΔΔCT^ was to normalize the gene. Primer sequences are presented in Table 1.

### 2.7. Total Protein Extraction and Western Blot Detection

As mentioned above, the detection of relevant proteins in this study is implemented by adopting western blot [21]. CNE2 cells were collected, and proteins were separated with Radio-Immunoprecipitation assay lysis buffer (Beyotime, Shanghai, China). The quantification of proteins was via the bicinchoninic acid kit (Merck, Germany). Electroblot of 30 *μ*g protein and 10% gel was onto polyvinylidene fluoride (PVDF) membrane and block was with 5% skim milk powder. Incubation of the membrane was with the following primary antibodies: Rabbit anti-human E-cadherin antibodies (1:800, ab40772), rabbit anti-human N-cadherin antibodies (1:1000, ab76011), anti-PTEN antibodies (1:1000, ab267787), and anti-*β*-actin antibodies (1:1000, ab8226). Horseradish peroxidase-labeled goat anti-rabbit secondary antibodies (1:5000, ab7090) were added, and continuous incubation was performed. All antibodies were purchased from Abcam (USA). Assessment and measurement of protein were implemented by adopting the electrogenerated chemiluminescence system (Beyotime).

### 2.8. The Luciferase Activity Assay

The luciferase activity assay was implemented on the grounds of the foregoing methods [22]. Cloning of mutant (WT) or wild-type (MUT) sequences of circSMARCA5 and PTEN 3′ UTR was into pmirGLO vector (Promega, USA). Co-transfection of the luciferase reporter plasmids with miR-582-3p-mimic and mimic-NC was into cells adopting Lipofectamine™ 2000 kit (Invitrogen). After 48 h of incubation, the analysis of the samples' luciferase activity was implemented by adopting the luciferase reporter assay system (Promega).

### 2.9. Statistical Analysis

All experiments were repeated at least three times and the display of data was as mean ± standard deviation. The adoption of SPSS 20.0 software was for statistical analysis, and the adoption of GraphPad Prism 7.0 software was to draw pictures. *T*-test and one-way analysis of variance were used for comparison between groups. *P* < 0.05 was accepted as indicative of distinct differences.

## 3. Results

### 3.1. CircSMARCA5 Is Elevated in NPC Tissues and Cells

The detection of circSMARCA5 in NPC tissues and cell lines was performed. The results illuminated that circSMARCA5 was overtly elevated in NPC tissues vs. the adjacent normal tissues (Figure 1(a)). Additionally, compared with HENE, NPC cell lines expressed circSMARCA5 at a higher level, among which the extreme elevation was presented in CNE2 cells and similar expression was presented in CNE1 and HONE1 cells (Figure 1(b)). The above data illuminated that circSMARCA5 might implicate NPC processes and was elevated in NPCs.

### 3.2. Silenced circSMARCA5 Restrains CNE2 Cell Advancement

In NPC cell lines, circSMARCA5 was most elevated in CNE2 cells, so the selection of CNE2 cells was for subsequent experiments. After transfection of si-circSMARCA5 and si-NC into CNE2 cells, circSMARCA5 was measured. The results elucidated circSMARCA5 in CNE2 cells was overtly declined after transfection with si-circSMARCA5 (Figure 2(a)). Cell advancement was evaluated and tested, clarifying that silenced circSMARCA5 distinctly restrained cell proliferation (Figure 2(b)-2(c)), migration (Figure 2(d)), and invasion (Figure 2(e)) after transfection with si-circSMARCA5. And consistent with that, silenced circSMARCA5 obviously promoted cell apoptosis (Figure 2(g)). Additionally, E-cadherin and N-cadherin were examined, illuminating that E-cadherin protein content was augmented while N-cadherin protein content was lessened after transfection with si-circ SMARCA5 (Figure 2(f)). The experimental results illustrated silenced circSMARCA5 was available to repress CNE2 cell advancement with the EMT process.

### 3.3. CircSMARCA5 Targets miR-582-3p

Antecedent studies have clarified that circRNA is available to stimulate or adsorb downstream miRNA to restrain miRNA's expression and function [23]. In the light of the predicting results of the starBase database, it was discovered that miR-582-3p was the target gene of circSMARCA5 (Figure 3(a)). The luciferase activity declined after co-transfection with miR-582-3p-mimic and circSMARCA5 WT, while the luciferase activity was almost unchanged after co-transfection with miR-582-3p-mimic and circSMARCA5 MUT (Figure 3(b)). Additionally, miR-582-3p was overtly strengthened after silencing circSMARCA5 (Figure 3(c)). In clinical tissues and cell samples of NPC, miR-582-3p was overtly declined vs. the adjacent normal tissues and HENE cells (Figure 3(d)-3(e)). Linear analysis results clarified that miR-582-3p was negatively linked with circSMARCA5 (Figure 3(f)). The above data illuminated that miR-582-3p was the target gene of circSMARCA5, and their expression patterns were opposite.

### 3.4. Elevated miR-582-3p Restrains CNE2 Cell Advancement

The biological function of miR-582-3p in NPC was detected. After separate transfection of miR-582-3p-NC and miR-582-3p-mimic into CNE2 cells, miR-582-3p's contents in CNE2 cells were determined. Data illustrated transfection with miR-582-3p-mimic augmented miR-582-3p (Figure 4(a)). After elevating miR-582-3p, cell proliferation (Figure 4(b)-4(c)), migration (Figure 4(d)), and invasion (Figure 4(e)) were all repressed; however, cell apoptosis rate was enhanced (Figure 4(g)). E-cadherin was augmented, while N-cadherin was lessened (Figure 4(f)). The experimental results clarified that elevated miR-582-3p was available to restrain CNE2 cell advancement.

### 3.5. Repressive miR-582-3p Turns around the Suppression of Silenced circSMARCA5 on NPC Cells

Co-transfection of si-circSMARCA5 and miR-582-3p-inhibitor was into CNE2 cells to explore their modulation on CNE2 cells. After transfection with si-circSMARCA5, miR-582-3p in CNE2 cells was distinctly strengthened, while miR-582-3p was overtly declined after co-transfection with miR-582-3p-inhibitor (Figure 5(a)). Silenced circSMARCA5 lowered cell proliferation (Figure 5(b)-5(c)), migration (Figure 5(d)), and invasion (Figure 5(e)) and increased cell apoptosis (Figure 5(g)). E-cadherin was augmented, while N-cadherin was lessened (Figure 5(f)). Nevertheless, this effect was blocked via transfection with miR-582-3p-inhibitor. These data elucidated that declined miR-582-3p was available to turn around the repression of silenced circSMARCA5 on NPC cell lines.

### 3.6. MiR-582-3p Targets PTEN

MiRNAs prevalently combine with the 3′ UTR of downstream mRNA and modulate its expression [24]. On the grounds of the forecast results of the starBase database, it was discovered that PTEN was miR-582-3p′s candidate target gene (Figure 6(a)). MiR-582-3p was available to bind to the 3′ UTR of PTEN and negatively modulated PTEN (Figure 6(b)). Additionally, transfection with miR-582-3p-mimic was available to lessened PTEN (Figures 6(c) and 6(d)). PTEN was elevated in NPC tissues and CNE2 cells vs. the adjacent normal tissues and HENE cells (*P* < 0.05) (Figure 6(e)-6(f)). Experimental data clarified that PTEN was the target gene of miR-582-3p, and miR-582-3p was available to target PTEN.

### 3.7. CircSMARCA5 Boosts the Malignant Phenotype of NPC via Modulating miR-582-3p/PTEN Axis

pcDNA-circSMARCA5 and si-PTEN were co-transfected into CNE2 cells to figure out the modulation of circSMARCA5 on PTEN. After transfection with pcDNA-circSMARCA5, PTEN in CNE2 cells was strengthened, while PTEN in CNE2 cells was weakened after co-transfection with pcDNA-circSMARCA5 and si-PTEN (Figure 7(a)-7(b)). Elevated circSMARCA5 enhanced cell proliferation (Figure 7(c)-7(d)), migration (Figure 7(e)), and invasion (Figure 7(f)) and attenuated cell apoptosis (Figure 7(h)). E-cadherin was lessened, while N-cadherin was augmented (Figure 7(g)). Nevertheless, these actions were blocked via transfection with si-PTEN. Additionally, linear analysis results illuminated that PTEN was positively associated with circSMARCA5 (Figure 7(i)). These data manifested elevated circSMARCA5 was available to elevate PTEN via restraining miR-582-3p, thereby boosting NPC's malignant phenotype.

## 4. Discussion

The incidence of NPC is regional with the extremely elevated incidence in the Asian population [25]. The disease has no specific symptoms at the early stage, while definite cases have entered the later stage, which rendered the possibility of cancer's distal metastasis to be higher and the risk of local recurrence is also superior [26, 27]. To better comprehend the mechanisms behind NPC occurrence and development, it is critical to ascertain reliable NPC markers. This research for the first time illuminated the regulatory association of circSMARCA5 with NPC, discovered circSMARCA5 was upper in NPC tissues and cell lines, suggesting that circSMARCA5 might be a biomarker for NPC diagnosis and treatment, and implicated in the development of elevated NPC.

Presently, circRNA in NPC is rarely explored. As reported, enhanced circMAN1A2 in NPC tissues is conducive to NPC diagnosis (AUC = 0.91) [28]. Elevated circ_0000285 is associated with tumor cell differentiation, tumor size, and distal metastasis and lymph node metastasis of NPC and can be adopted as an independent prognostic index of NPC [29]. Circ_0066755 is overtly expressed in NPC patients' plasma and tissues and is positively linked with tumor progression. Additionally, circ_0066755 in plasma is extremely consistent with MRI diagnosis in NPC diagnosis, and blood samples are available to be obtained more easily via a minor invasive sampling process, which makes circ_0066755 in plasma a promising diagnostic NPC index [30]. SMARCA5, also known as SNF2H, derived from SWI/SNF with matrix association, is an actin-dependent regulator of chromatin with helicase and ATP enzymatic activities and modulates and reshapes chromatin [31]. CircSMARCA5 is generated via the SMARCA5 gene of exons 15 and 16. Researches have manifested that circSMARCA5 is linked with cancer's clinicopathologic features. For instance, circSMARCA5 is restrained in HCC. Additionally, declined circSMARCA5 in HCC is negatively associated with overall survival and relapse-free survival after hepatectomy, indicating that circSMARCA5 restrained the advancement of HCC as a tumor suppressor vs. the adjacent normal tissues [32]. CircSMARCA5 is declined in cancers like multiple myeloma, GC, non-small cell lung cancer, and intrahepatic cholangiocarcinoma, and elevated circSMARCA5 is an independent risk factor for prolongation of overall survival and good prognosis [33, 34]. Nevertheless, circSMARCA5 is strengthened in PCa and CC, which boosts cell advancement, indicating that circSMARCA5 might perform as a cancer-promoting gene in cancer development [35]. The controversial expression pattern and action of circSMARCA5 in cancer might be attributed to molecular diversity in tumorigenesis [36]. This article firstly put forward and verified that circSMARCA5 was distinctly elevated in NPCs. The experimental results of this study elucidated silenced circSMARCA5 was available to lessen CNE2 cell advancement.

MiR-582-3p, as a kind of miRNAs, is available to adsorb and combine with upstream circRNA and modulates cancer's development. Studies have discovered that circEYA1 is available to repress miR-582-3p, elevate C-X-C motif chemokine ligand 14, and restrain cervical adenocarcinoma tumors' occurrence [37]. MiR-582-3p in combination with miR-582-5p is available to suppress PCa to bone metastasis via restraining TGF-*β* signal transduction [38]. MiR-582-3p is available to target DLX2 to repress HCC's development, and miR-582-3p in HCC cell line Huh-7 and HCCLM3 is silenced vs. the normal hepatocytes [39]. Although the role of miR-582-3p in NPCs has been previously reported, we demonstrate for the first time that circSMARCA5 provides a role in NPC biology via sponging miR-582-3p. MiR-582-3p was declined in NPC tissues and cell lines. Combined with the analysis and prediction of bioinformatic data and the luciferase activity assay results, this study testified the existence of a binding site of miR-582-3p with circSMARCA5, which was available to adsorb and negatively modulate miR-582-3p. The results of functional experiments indicated elevated miR-582-3p restrained CNE2 cell advancement, while repressive miR-582-3p was available to block the therapeutic action of silenced circSMARCA5. These results clarified that miR-582-3p was available to silence the process of NPC and accelerate cancer cell apoptosis.

PTEN, located on chromosome 10, is first identified in 1990 as a tumor suppressor gene and a negative regulator of the PI3K/Akt/mTOR pathway [40]. The gene of encoding PTEN is structurally composed of nine exons, which participate in the formation of the avail of dual functional 4,3-amino acid protein lipids and protein phosphatases [41]. PTEN is available to exert a tumor suppressor role via sustaining chromosomal stability and controls DNA repair protein RAD51 to stimulate DNA repair, while silenced PTEN is available to lead to genomic instability and repress homologous recombination [42]. Based on the distinct role of PTEN in modulating the PI3K/Akt/mTOR pathway and the pathway in cell survival and proliferation, in numerous researches, PTEN's action in cancer is explored, such as LC [43], colon cancer [44], bladder cancer [45], etc. PTEN's action in NPC has also been figured out. Placental-specific protein 1 is available to accelerate NPC cell proliferation and migration and enhance cancer cell invasion ability via the Furin/NICD/PTEN pathway [46]. MiR-214 mediates NPC cell viability and apoptosis via targeting WWOX and PTEN [47]. PTEN is available to repress small interfering RNAs, thereby boosting NPC's occurrence and advancement [48]. This article further explored the association of PTEN with NPCs. In the light of the prediction of bioinformatic tools and the verification of the luciferase activity assay, it was discovered that PTEN was the target gene of miR-582-3p, they were provided with binding sites, and miR-582-3p negatively modulated PTEN, which was also elevated in NPC tissues and cell lines. The above experimental results illuminated PTEN implicated in the modulation of NPC and elevated the illness.

Several studies have shown that Chinese herbal medicine plays an important role in the prevention and treatment of some cancers. For instance, the Chinese herbal mixture, such as Zeng-Sheng-Ping, has been shown to inhibit tumor progression in lung cancer (PMID: 15021904). With the deepening of research on traditional Chinese medicine, their mechanism of action has been gradually discovered. For example, Samsoeum efficiently induces cancer cell death via apoptosis and autophagy through regulating Akt/mTOR and JNK signaling pathways (PMID: 24053190). Qing Yan Li Ge Tang could induce autophagic cell death in NPC cells through the PI3K/Akt/mTOR pathway (PMID:34765012). Nevertheless, whether circSMARCA5/miR-582-3p/PTEN axis could be used as the target of traditional Chinese medicine for the treatment of NPC needs to be further verified.

In brief, the results of the research have elucidated that circSMARCA5 is available to modulate CNE2 cell advancement via miR-582-3p/PTEN axis. CircSMARCA5 is expected to be a new candidate biomarker for NPC prevention and diagnosis and offers a theoretical foundation for subsequent experiments. Furthermore, several limitations are presented in the study. In the research, circSMARCA5 modulates NPC via miR-582-3p/PTEN, but this pathway's specific curative mechanism remains to be further explored. Additionally, clinical trials have not been carried out in the research, so the treatment outcome of patients fails to be assessed. Consequently, more complete experiments and analyses are required for subsequent experiments.

## Figures and Tables

**Figure 1:** CircSMARCA5 is elevated in NPC tissues and cells. (a) RT-qPCR test of circSMARCA5 in NPC tissues and adjacent normal tissues; (b) RT-qPCR examination of circSMARCA5 in human embryonic nasopharyngeal epithelial cell HENE and NPC cell lines CNE1, HONE1, and CNE2. ^*∗*^*P* < 0.05.

**Figure 2:** Silenced circSMARCA5 restrains CNE2 cell advancement. (a) RT-qPCR examination of circSMARCA5 after transfection with si-circSMARCA5; (b) MTT assay test of the impact of silenced circSMARCA5 on CNE2 cell proliferation; (c) cell colony formation assay examination of CNE2 cell proliferation after silencing circSMARCA5; (d, e) Transwell assay test of CNE2 cell migration and invasion after silencing circSMARCA5; (f) western blot examination of E-cadherin and N-cadherin after silencing circSMARCA5; (g) flow cytometry test of CNE2 cell apoptosis rate after silencing circSMARCA5. All experiments were repeated three times, ^*∗*^*P* < 0.05.

**Figure 3:** CircSMARCA5 targets miR-582-3p. (a) Through https://starbase.sysu.edu.cn/ forecast of the combination domain of miR-582-3p and circSMARCA5; (b) luciferase activity assay verification of the targeting of circSMARCA5 with miR-582-3p; (c) RT-qPCR detection of miR-370-3p after silencing circSMARCA5; (d, e) RT-qPCR examination of miR-582-3p in NPC tissues and cell lines. (f) circSMARCA5 was negatively associated with miR-582-3p. All experiments were repeated three times, ^*∗*^*P* < 0.05.

**Figure 4:** Elevated miR-582-3p represses CNE2 cell advancement. (a) After transfection of miR-582-3p-mimic into CNE2 cells, RT-qPCR test of miR-582-3p; (b) MTT assay examination of cell proliferation; (c) cell colony formation assay test of cell proliferation; (d, e) Transwell assay test of cell migration and invasion ability; (f) western blot examination of E-cadherin and N-cadherin; (g) flow cytometry test of cell apoptosis. All experiments were repeated three times, ^*∗*^*P* < 0.05.

**Figure 5:** Suppressive miR-582-3p turns around the repression of silenced circSMARCA5 on NPC cells (a) Co-transfection of si-circSMARCA5 and miR-582-3p-inhibitor was into CNE2 cells, and RT-qPCR test of miR-582-3p; (b) MTT assay examination of cell proliferation; (c) cell colony formation assay test of cell proliferation; (d, e) Transwell assay examination of cell migration and invasion; (f) western blot test of E-cadherin and N-cadherin; (g) flow cytometry examination of cell apoptosis. All experiments were repeated three times, ^*∗*^*P* < 0.05.

**Figure 6:** MiR-582-3p targets PTEN. (a) The binding domain of miR-582-3p with PTEN; (b) luciferase activity assay verification of the targeting of miR-582-3p and PTEN; (c, d) RT-qPCR and western blot detection of targeted regulation of miR-582-3p with PTEN; (e, f) PTEN in NPC tissues and cell lines. All experiments were repeated three times, ^*∗*^*P* < 0.05.

**Figure 7:** CircSMARCA5 elevates NPCS via modulating miR-582-3p/PTEN axis. (a, b) After co-transfection of si-PTEN and pcDNA 3.1-circSMARCA5 into CNE2 cells, RT-qPCR and western blot examination of PTEN; (c) MTT assay test of cell proliferation; (d) cell colony formation assay examination of cell proliferation; (e, f) Transwell assay test of cell migration and invasion; (g) western blot test of E-cadherin and N-cadherin; (h) fow cytometry examination of cell apoptosis; (i) linear calculation analysis of the relevance of PTEN with circS MARCA5. All experiments were repeated three times, ^*∗*^*P* < 0.05.

**Table 1:** Primer sequences.

Genes		Primer sequences
MiR-582-3p	F:	GCCGAGTAACTGGTTGAACA
	R:	CTCAACTGGTGTCGTGGA

U6	F:	CTCGCTTCGGCAGCACA
	R:	AACGCTTCACGAATTTGCGT

CircSMARCA5	F:	CTCCAAGATGGGCGAAAG
	R:	TGTGTTGCTCCATGTCTAATCA

PTEN	F:	CTTACAGTTGGGCCCTGTACCATCC
	R:	TTTGATGCTGCCGGTAAACTCCACT

*β*-actin	F:	CCTCTCCCAAGTCCACACAG
	R:	GGGCACGAAGGCTCATCATT

## Data Availability

The data that support the findings of this study are available from the corresponding author upon request.
